# A Pyramid Architecture-Based Deep Learning Framework for Breast Cancer Detection

**DOI:** 10.1155/2021/2567202

**Published:** 2021-10-01

**Authors:** Dong Sui, Weifeng Liu, Jing Chen, Chunxiao Zhao, Xiaoxuan Ma, Maozu Guo, Zhaofeng Tian

**Affiliations:** ^1^School of Electrical and Information Engineering, Beijing University of Civil Engineering and Architecture, Beijing 100044, China; ^2^Department of Laboratory and Diagnosis, Changhai Hospital, Navy Medical University, Shanghai 200433, China

## Abstract

Breast cancer diagnosis is a critical step in clinical decision making, and this is achieved by making a pathological slide and gives a decision by the doctors, which is the method of final decision making for cancer diagnosis. Traditionally, the doctors usually check the pathological images by visual inspection under the microscope. Whole-slide images (WSIs) have supported the state-of-the-art diagnosis results and have been admitted as the gold standard clinically. However, this task is time-consuming and labour-intensive, and all of these limitations make low efficiency in decision making. Medical image processing protocols have been used for this task during the last decades and have obtained satisfactory results under some conditions; especially in the deep learning era, it has exhibited the advantages than those in the shallow learning period. In this paper, we proposed a novel breast cancer region mining framework based on deep pyramid architecture from multilevel and multiscale breast pathological WSIs. We incorporate the tissue- and cell-level information together and integrate these into a LSTM model for the final sequence modelling, which successfully keeps the WSIs' integration and is not mentioned by the prevalence frameworks. The experiment results demonstrated that our proposed framework greatly improved the detection accuracy than that only using tissue-level information.

## 1. Introduction

Breast cancer is the leading death cause among women all over the world [1]. Great progresses of microscopic imaging make digital pathology come into the whole-slide image (WSI) stage. These techniques allow a WSI image (a whole-slide image at 40x magnification is about 2 GB) to be stored, served, and viewed in multiscale, multiview, and multilevel than the light microscopy. In this context, modern precision medicine approaches require careful diagnostic with personality and precision survival prediction for each case so as to tailor suitable therapy protocol [2]. A straight diagnostic protocol of breast cancer is the interpretation of digital pathology slides, which used to be a time-consuming and labour-intensity pathway for manual interpretation with significant inter- and introobserver variability [3]. The computer-aided digital pathology analysis combines the image processing technique that opens the door to automatically depicting the pathology slides with a more objective and quantitative way [4]. Over these decades, due to the breakthroughs in Artificial Intelligence (AI), it allows computers to reach the state of the art in many vision-based tasks, better than human counterparts for specific tasks, especially in the field of medical image processing [5].

Clinically, pathological analyses on axilla lymph nodes can indicate the original, spread, and metastasis of breast cancer; furthermore, the pathological changes in axilla lymph nodes are a critical factor for prognostic evaluation [6]. However, pathological image analysis in lymph nodes in tissue level is usually time-consuming and prone to subjective variances. In addition, small metastases such as isolated tumor cell clusters (ITCs) are a small region with few cells and difficult to detect or missed [7]. Based on these merits, there are great demands of automated breast cancer detection frameworks for improving the robustness and precision of the decision making [4]. WSIs excited the development of quantitative histopathology analysis, which can now capture nuclear and tissue architecture from different levels and scales [8, 9]. Furthermore, cell-level analysis based on cell shape, nuclear morphology, and cytoplasm distribution is crucial for the tumor grading and reorganization [10]. It has been reported that many cell analysis frameworks give the possibility for incorporating with cell-level information to analyze the multiscale pathological image [5, 11].

In this paradigm, many deep learning-based metastasis detection methods have been proposed and achieved excellent results at the challenges in MICCAI and ISBI from 2016~2020 [12, 13]. A consistent evaluation of digital pathology analysis protocols for breast cancer diagnosis with accuracy and efficiency was performed; all of these successes are dependent on the proper designing and integrating exiting pipeline by using transfer learning. In this way, researchers can reduce the risk of cancer patient and slide misidentification; furthermore, tissue loss and damage can be better fixed to facilitate covering the gaps among pathology laboratories and clinical primary diagnosis [14]. Thus, the most important advantage of WSIs is that the researchers can apply deep learning-based methods in the diagnostic workflow. However, most of these frameworks mainly focus on tissue level in the WSIs and cannot depict the details of cell-level information.

## 2. Related Work

Detection of the suspected tumor region, characterization of tumor subtype, and quantification of tumor invasive extent are the critical procedure in breast cancer diagnostic. In deep learning context, CNN is employed for breast cancer WSI patch classification, in which the CNN model uses manually annotated labels for training and gets ideal results [15]. Cruz-Roa et al. proposed a deep learning pipeline that is pretrained using image net for distinguishing the benign and malignant breast cancer; at the same time, some data augmentation methods have been adopted to prevent overfitting [16]. Lymph node metastasis is the most suitable background for AI algorithm application; Liu et al. and Steiner et al. proposed a challenge competition and establish a testbed for breast cancer diagnosis; the comparison results exhibited great superiority for the deep learning-based method than the pathologist achievement [17, 18]. On the other hand, tumor histologic grading and invasive tumor characterization can give a deep inspection for breast cancer prognostic evaluation. But cell-level and tissue-level feature identification used to be a laborious task, such as the tubular formation and mitotic cell analysis, which are important prognostic factors that were mined by using manual operation, and the labour-intensive nature of mitotic counting can lead to discordance.

Some shallow learning methods have achieved remarkable results on this paradigm [19, 20]; recently, deep learning methods have shown their excellent performance on this task [21–23]. For the early achievement, Rexhepaj et al. proposed a nuclear detection algorithm to quantify IHC staining cell for protein expression and get a correlation of 0.9 with manual counting [24]. Nonetheless, this method has not achieved the state of the art at that time; the subsequent work shows that the deep learning-based method can help improve the level of concordance among human pathologists [24]. Romo et al.'s team employed a CNN model to detect tubule nuclei and use this information for Oncotype DX risk category [25]. Veta et al. propose a framework based on non-CNN model to perform cell nucleus detection and segmentation jointly for the cell morphological analysis [22, 25]. Biomarker finding is another element that related with diagnosis of breast cancer. More recently, WSI-based biomarker detection is becoming a prominent pathway for tumor evaluation directly using image information. Couture et al. introduced a deep learning-based multimodule framework for ER status prediction and get the accuracy up to 84% [26]. Shamai et al. implemented a deep learning pipeline with less data of 19 biomarkers, and within the subgroup, they get the 92% accuracy of confidence score [27]. Image of aspiration biopsy was also employed to mining malignant and benign tumors by fitting cellular features with machine learning paradigm [28]. The conditional GAN model is a promising pathway of image data augmentation for the deep model training. Sahiner et al.'s works supported the application of GANs to boost the training phase to optimize tumor classification [29].

The morphological features extracted from the breast cancer WSIs are known to be valuable for the prognosis evaluation. Veta et al. use breast cancer microarray data and nuclear handcraft features to construct a general model for patients' prognosis evaluation, and their research open a window for the possible direction of tumor prognosis analysis by multimodule feature fusion [19, 20]. As a standard deep learning model, CNN can extract multiple-level features to represent the tumor region; Yuan proposed a CNN-based model to analyze the lymphocyte spatial distribution for classifying different tumors in WSIs [30]. In addition, the spatial relationship is also used for cell morphology analysis, tumor detection, and prognosis evaluation, but there are still few researches that focus on multilevel and multiscale information. In this paper, we proposed an open and multitask framework for tumor detection and grading; we also concern some spatial information and multilevel fusion features to depict the hidden relationship between tumor statues and information from each level.

## 3. Materials and Methods

### 3.1. Datasets

For the framework construction, we use Camelyon 2017 data set for the tissue-level network training and TIM 2015 data set for cell-level detection network training, respectively [7, 31]. Although there are many other data sets for the cancer region detection of breast cancer, we still choose the Camelyon 2017 data set for the evaluation; this is because of the restriction of data scale and the processing ability of our hardware platform.  Figure 1 shows the details of the two data samples. For the framework construction, we use the Camelyon 2017 data set for the tissue- level network training and the TIM 2015 data set for cell-level detection network training, respectively. The TIM2015 data set can be found at http://haeckel.case.edu/data/TMI2015.tgz, and the Camelyon 2017 data set can be found at https://camelyon17.grand-challenge.org/.

The Camelyon 2017 data set is a multilevel WSI data set including patients from different medical centers and up to 500 slides; for the network training, we manually selected 100 slides for this task. The glass slides were digitized by whole-slide scanners with a pixel size of 0.23 to 0.26 *μ*m, respectively. The WSI is a multiple-resolution and multiple-level images that is about 1 × 10^5^ by 2 × 10^5^ pixels at the highest resolution level. The whole WSI contains 10 resolution levels; each consecutive level doubled the pixel size in both directions and halved the pixel in each dimension; in addition, the file size of a WSI with 10 levels is about 2~4 GB which varies depending on the scanner and tissue anatomy structure of the input image. The scanned images were converted into standard multiresolution TIFF image files according to open slide standard [7].

The TMI 2015 data set is also H&E-stained histopathological images, which were obtained from digitized glass slides corresponding to 49 lymph node-negative and estrogen receptor-positive breast cancer (LN-, ER+ BC) patients at Case Western Reserve University. The size of each image is about 2200 × 2200 pixels, and there are about 1500 nuclei in each image [31].

### 3.2. Pathological Region Generation

For the training of the pyramid deconvolution network, balance of the training sample is a critical problem, but in this data set, the tumor types are unbalance in different tumor stages. For this situation, we adopted the deep convolution generative adversarial networks (DCGAN) for boosting the tumor region patches and extended the origin patch set into an expanded edition. Under this situation, the data unbalance can be addressed as a data generation problem from the existing classes, so as to promote the balance of the training data.  Figure 2 shows the details of the pathological image generation process for the microregion of breast cancer.

### 3.3. Whole-Slide Image Preprocessing

In this paper, we employed two data sets, part of Camelyon 2017 and the TMI 2015 from breast cancer tissue section slide. For WSIs of Camelyon 2017, we extracted the slide area on each level by OTSU algorithm. Following this step, we split the original image into small patches with the same size at each scale. At the same time, we transform the counter label of Camelyon 2017 into mask and perform the same manipulation with its WSI image at each level. Concerning the image quality, we chose a commonly used color equalization to reduce the effect of unequalization and uneven illumination of original WSI staining [32].

Because the cancer regions in the Camelyon 2017 data set only cover a small region in the WSI slides, this led to an unbalance situation for the deep model training. We adopt some data augmentation methods to merge the gap, such as random cropping, colour jittering, scaling, and rotation. For some class, we use deep convolution generative adversarial networks (DCGAN) for boosting the tumor region patches; finally, we extended the origin patch set into an expanded edition.

For the TIM2015 data set [31], this data set is used for training and evaluating a cell detection model; the original data was labeled by using a binding box; for convenience and application, we transform the binding box into a point label by making an average position through the four coordinates of the binding box. Then, following our proposed method, we fill the dot label with Gaussian kernel for the cell mask generation, and at last, we constructed the final training set for cell-level analysis pipeline.

### 3.4. Framework Architecture and Network Design

In this paper, we construct a multilevel and multiscale tumor region detection and segmentation framework for breast cancer. As it is shown in Figure 3, the WSIs are stored into a multiple-level pyramid structure with 10 levels; the user can zoom into any level and depict the details to perform diagnosing tasks. For this situation, we divided the total framework into two levels of tumor analysis procedure pipeline, in the tissue level and cell level, we adopt the same network backbone architecture derived from the DeconvNet (see Figure 4), and some parameter settings are also changed according to the input image. In the following part, we will introduce the details of our framework in the tissue level and cell level, respectively.

The aim of the tissue level is to get the tumor region according to the labeled mask so as to assign the TNM stage of WSI. As shown in Figure 4, the tissue level and cell level share the same basic network. They are all based on DeconvNet which consists of the stacked convolution layers, max-pooling layers, and deconvolution layers. In the front three blocks, max-pooling layers are followed with convolution layers, and ReLU activation layer and convolution layer which form deconvolution layers are followed with upsampling layers which are followed by the last three blocks. Finally, a convolution layer was used to replace fully convolutional layers in the end of the network in order to obtain a density map. Totally speaking, 3 × 3 kernel size, ReLU activation, Mean Squared Error (MSE) loss function, and Adam optimizer were used in all network structures. In order to handle different tasks, the basic network was fine-tuned. As shown in Figure 2, the fully connected layer was connected to the last convolution layer to get confidence result of patch binary classification. With characteristic of DeconvNet, images of any size can be input. However, in actual application, images with the dimensions reduction were used to avoid cutting the edge of the output density map.

For the high-resolution WSI images, the content is usually up to 2 GB for a single image, and the tumor region locates at somewhere in the whole slide. For a large image, the network has to be trained on the image patches generated from the ground scale. In order to keep the patch sequencing, we proposed a LSTM-CFCN-based model for the segmentation task. In this model, the stacked channel FCN is for the patch feature encoding and the LSTM model is used to merge these patches into a large image from these FCN encoded patches; more details are illustrated in Figure 5. In this part, the cancer region in the training data set is labelled by using a mask; the channel FCN is used to estimate the density map of a tumor region in each sequential patch; and LSTM block is used to combine the detected result into an integrated figure. From this point of view, the tumor density map is predicted by the deconvolution part, and a Euclidean distance is used for measuring the difference between the generated density map and the ground truth. And the loss function is defined as follows:

(1) $$\begin{array}{c} L_{t}=\frac{1}{2N}\overset{N}{\underset{i=1}{\sum }}\overset{p}{\underset{p=1}{\sum }}{\left\|F_{i}\left(p;\Theta_{\text{CFCN}}\right)-F_{i}^{0}\left(p\right)\right\|}_{2}^{2}, \end{array}$$

where *N* is the batch size and *F*_*i*_(*p*) is the probability of tumor at pixel *p* in the *i*th sequential patch. For some situation in low level of WSI, the global tumor region is generated from several sequential image patches; the integration is learned by the LSTM block. So, the total loss function includes the basic tumor segmentation part and the LSTM residual part. The final result is a sum of the two parts:

(2) $$\begin{array}{c} T_{i}=R\left(F_{i};ϒ,\Psi \right)+\overset{P}{\underset{p=1}{\sum }}F_{i}\left(p\right), \end{array}$$

where *R*(*F*_*i*_; *ϒ*, Ψ) is the residual count, *F_i_* is the estimated heat map from patch *i*, *ϒ* is the parameter of LSTM, and Ψ is the fully connected layer's parameter. The whole-slide tumor detection loss function is defined as

(3) $$\begin{array}{c} L_{\text{lstm}}=\frac{1}{2N}\overset{N}{\underset{i=1}{\sum }}{\left(T_{i}-T_{i}^{0}\right)}^{2}, \end{array}$$

where *T*_*i*_^0^ is the ground truth in the *i*th image patch and *T*_*i*_ is the learned tumor region. In this way, the total loss function for the multiple-scale LSTM-CFCN is defined as

(4) $$\begin{array}{c} L=L_{t}+\alpha L_{\text{lstm}}, \end{array}$$

where alpha is a weight parameter of the LSTM residue and to be tuned for the suitable accuracy. At the same time, the tumor detection is trained with fewer parameters to achieve a better training process. In the framework, the Adam optimizer and backpropagation are used to optimize the loss function *L* for different scenes.

### 3.5. Tissue-Level Pyramid-DeconvNet

In the tissue level, conventional deep learning methods usually take amount of time and space to handle all the small patches. In order to overcome this obstacle, we introduce a flexible automatic decision method based on the pyramid deconvolution networks, which can target the RoIs (Region of Interest) quickly with higher accuracy. We first cast the problem as a supervised learning problem that tries to learn a mapping between a patch *I*_*l*_(*x*) and a density map *D*_*l*_(*x*), denoted as*F*_*l*_ : *I*_*l*_(*x*)⟶*D*_*l*_(*x*) which, (*I*_*l*_ ∈ *R*^*m*×*n*^, *D*_*l*_ ∈ *R*^*m*×*n*^) in layer *l* and obtained different weights *w*_*l*_ and biases *b*_*l*_. Then, we fixed *w*_*l*_ and *b*_*l*_ to train the last fully connected layer for classification *C*_*l*_(*w*_*l*_, *b*_*l*_, *w*_*l*_^*fc*^, *b*_*l*_^*fc*^). Utilizing a tree-like searching protocol, networks in layer *l* will test their layer separately with *C*_*l*_ and obtained the classification confidence of cancer *C*(*x*). RoI prediction probability was compared with threshold *t*. If we find RoI, we introduce location code information, short for LCI, which is a series of continuous coding to represent the position of each RoI and find the coordinates and LCIs of next layer *l* − 1. Loop until we reach the top layer of cell level. Details are shown in Algorithm 1.

### 3.6. Cell-Level DeconvNet

In the small tumor region of the WSI images, it even contains few illness cells. The cell-encoding information is obtained for better judgment of small tumor areas, such as micro and ITC. For the tumor region affirmative, we introduce a cell-level DeconvNet. The basic network is a DeconvNet with a NMS layer embedded to the last convolution layer. After training, the proposed network with patches and their mask images were filled with Gaussian kernels with Equation ((1)):

(5) $$\begin{array}{c} P\left(x\right)=\frac{1}{{\left(2\pi \right)}^{D/2}{\left|\Sigma \right|}^{1/2}}\exp\left\{-\frac{1}{2}{\left(x-\mu \right)}^{T}\Sigma^{-1}\left(x-\mu \right)\right\}. \end{array}$$

Density maps which consist of 0-1 float values of each layer were obtained. After that, NMS was employed to get the accuracy of each cancer cell. And then, we view the value of detection count results as cancer cell counting results and cluster the detected points to form the region of cancer area. As shown in Figure 3, a Nonmaximum Suppression (NMS) algorithm was connected to the final layer to get the position of each cell and obtain the result of cancer cell counting and region area. In this way, the small region such as ITC and micro are detected by using cell-level screening.

### 3.7. Cancer Region Generation

Through tissue-level detection method, if Algorithm 1 breaks with layer number larger than two, the WSI is negative. And macro areas and large size of microareas were detected if the total area of connected RoI patches in layer two were larger than the threshold of the area in the TNM staging system. And then, cell level determined the areas of micro or ITC, which were passed to a cancer cell detector to obtain the location and number of cancer cells. The size of cancer areas and the number of cancer cells were breast cancer detection standard to classify the images according to the TNM system.

### 3.8. Evaluation Methods

For the tumor segmentation, we evaluated the segmentation performance by using the tradition method of image segmentation. The results of our pipeline are reported in terms of recall, precision, and *F*_1_-measure value, as follows:

(6) $$\begin{array}{c} \text{Recall}=\frac{\text{TP}}{\text{TP}+\text{FN}},\\ \text{Precision}=\frac{\text{TP}}{\text{TP}+\text{FP}},\\ F_{1}=\frac{2PR}{P+R}. \end{array}$$

For the evaluation, we choose the intersection over union (IoU) metric and Jaccard index to quantify the percent overlap between the target mask and the framework prediction output results. The Jaccard similarity coefficient of the segmentation result and the original labelled mask is expressed as

(7) $$\begin{array}{c} \text{Jaccard}\left(S,M\right)=\frac{\left|\text{intersection}\left(S,M\right)\right|}{\left|\text{union}\left(S,M\right)\right|}, \end{array}$$

where |∗| represents the cardinal of set ∗. The Jaccard index can also be expressed in terms of True Positives (TP), False Positives (FP), and False Negatives (FN) as

(8) $$\begin{array}{c} \text{IoU}=\frac{\text{TP}}{\text{TP}+\text{FP}+\text{FN}}. \end{array}$$

## 4. Results and Discussion

### 4.1. Network Training

All experiments and test bed are carried out on Intel Core (TM) i9, 12 cores, 2.90 GHz processor with 32 GB of RAM and a NVIDIA GeForce GTX 2080Ti Graphics Processor Unit. The software implementation is performed using CUDA10.0, CuDNN8.5, and Pytorch1.5.

The proposed models have been tested on the Camelyon 2017 data sets; in this part, we divided each data set into two parts, 70% and 30% for training and testing. We kept the same parameters in all FCN blocks to make sure the network stability. For making sure the cells in LSTM model, we performed several tests about the cell number; finally, we choose the *N* with 10 cells. The training epoch generally kept at 3000 for the pathological images. In the training processes, random sampling and truncated back propagation are employed for handling the huge image data and LSTM model tuning. Adam optimizer is used in these models with 1*e*-3 and final learning rate with 1*e*-5, and the learning rate is reduced by an equal step in each epoch until the final learning rate is reached.

### 4.2. Results of Tumor Region Detection

In this paper, we proposed a multiple-level CFCN-based framework for the tumor region detection in breast cancer WSI image data set. The final aim is to combine the pyramid information from different image scales to ensure the accuracy of final segmentation results. In this part, we choose several tissue-level and cell-level information for the segmentation task and get a relative satisfactory decision on the test set.

The segmentation results of our proposed framework are shown in Figure 6. For the tissue-level detection, we applied the framework to carry out the tumor region detection task on the Camelyon 2017 data set. Here, we selected some segmentation result as the final tissue-level detection; in Figure 6, the heat maps (b) and (f) exhibit the tumor region in the WSI slides. For the segmentation details, (d) and (h) are the partial details of the segmentation result on the WSIs; it can depict that our proposed framework can distinguish the tumor region and normal region clearly in the testing set.

For the comparisons, we choose some state-of-the-art methods such as FCN and U-Net as the test bed for the final method evaluation. In tissue-level segmentation, we compared our proposed method with the abovementioned methods; results are shown in Table 1; for the normal region in WSIs, our proposed framework gets the highest accuracy compared with the traditional methods. In addition, U-Net usually takes the priority position in medical image processing especially on segmentation task, but the U-net model cannot depict the level-wise information. In our framework, we use both cell-level and tissue-level information for the final decision and get a higher accurate result. Micro and ITCs are small regions that contain few cancer cells with unstable variability in morphology, usually existing at an unstable statute in the whole slide. All of these induced the low accuracy of detection and segmentation. In this situation, our framework still catches the better results for some fixed situation.

To refine the segmentation results, we combined the cell-level information into the framework and make sure the segmented tumor region contains multilevel information. Especially for the micro and ITC regions, the cell-level information can indicate the existence of small tumor regions even without screening by tissue-level scans. For cell-level information incorporation, we can see that it can improve the detection result, Table 1 shows the detection results by employing cell-level and tissue-level information, and there is a certain improvement on detection accuracy.  Figure 7 shows the segmentation result by using different methods; it can be addressed; our proposed method can greatly improve the segmentation result compared with FCN and U-Net.

## 5. Conclusions

In this paper, we propose an automatic cancer lesion detection approach using pyramid deconvolution network (PDN) for multilevel and multiscale H&E-stained breast pathological WSIs. In this framework, we integrate tissue- and cell-level information for the cancerous region detection and segmentation, which is neglected by state-of-the-art methods. The results demonstrated that our workflow greatly improved the performance compared with those only using tissue-level information. The comparison results showed our framework can get better accuracy on the same testing data set. In the future, our aim will focus on multiscale feature extraction and fine-tuning the new representation network for improving the detection and segmentation performance.

## Figures and Tables

**Figure 1:** Data set in this paper. (a) Is the Camelyon 2017 whole-slide images [7]; (b) is the TMI 2015 data set from Xu et al. [31].

**Figure 2:** GAN model for pathological image generation.

**Figure 3:** The scheme of pyramid deconvolution network framework for breast cancer detection.

**Figure 4:** The backbone network architecture of the DeconvNet. We make a slight change on kernel size and stride for different input image scales.

**Figure 5:** Long short-term memory enhanced channeled fully convolutional network pipeline with a dimension shuffle layer.

**Figure 6:** Pathological images and their detection results. The subimages (a), (c), (e), and (g) are the original pathological images; (b) and (f) are the heat maps generated from our framework.

**Figure 7:** Comparisons of the segmentation results among different methods. (a–d) Are different views of the WSIs; from 1 to 4 are the segmentation results of original image, FCN, U-net, and our proposed method.

**Algorithm 1:** Tissue-level pathological RoI extraction.

**Table 1:** Comparison results of different methods.

Methods/accuracy	Normal (%)	Macro (%)	Micro (%)	ITCs (%)	Average (tumor, %)
FCN	64.3	61.1	53.6	17.3	44
U-Net	77.8	67.1	55.2	21.2	47.83
Ours	80.1	73.6	57.7	20.6	50.63
FCN + cell detection	68.7	64.7	54.2	14.1	44.33
U − Net + cell detection	79.6	70.1	58.4	23.1	50.53
Ours + cell detection	85.3	74.3	60.1	24.6	53

## Data Availability

The pathological image data used to support the findings of this study are available from the corresponding author upon request.
